# Sport Resource Classification Algorithm for Health Promotion Based on Cloud Computing: Rhythmic Gymnastics' Example

This article has been retracted.

**DOI:** 10.1155/2022/2587169

**Published:** 2022-07-30

**Authors:** Tairan Zhang, Qing Han, Zhenji Zhang

**Affiliations:** ^1^School of Economics and Management, Beijing Jiaotong University, Beijing 100044, China; ^2^College of Physical Education and Sports, Beijing Normal University, Beijing 100875, China

## Abstract

In the processing of rhythmic gymnastics resources, there are inefficiency problems such as confusion of teaching resources and lack of individuation. To improve the health access to teaching resource data, such as videos and documents, this study proposes a cloud computing-based personalized rhythmic gymnastics teaching resource classification algorithm for health promotion. First, personalized rhythmic gymnastics teaching resource database is designed based on cloud computing technology, and the teaching resources in the database are preprocessed to obtain a meta-sample set. Then, the characteristics of teaching resources are selected by the information acquisition method, and a vector space model is established to calculate the similarity of teaching resources. Finally, the distance-weighted k-NN method is used to classify the teaching resources for health promotion. The experimental results show that the classification accuracy of the proposed algorithm is high, the recall rate is high, and the F-measure value is high, which verifies the effectiveness of the algorithm.

## 1. Introduction

Rhythmic gymnastics for health promotion ([1], p.977) has entered the field of physical education in universities for many years. Its combination of dance, gymnastics, and music is very in line with the needs of female college students for fitness and body shaping. Therefore, it is deeply loved by female college students. However, the current college rhythmic gymnastics for health promotion teaching has been using traditional teaching methods ([2], p.22), which has been challenging to meet the needs of the rapid development of today's society. How to effectively improve the effectiveness of rhythmic gymnastics for health promotion classroom teaching has become an urgent problem in college rhythmic gymnastics for health promotion teaching ([3], p.15). Information-based teaching methods have been widely used in colleges and universities, which can significantly improve the teaching efficiency of rhythmic gymnastics for health promotion and promote the sharing and construction of rhythmic gymnastics for health promotion resources ([4], p.147). In addition, this teaching method can improve students' interest in learning and the quality of classroom teaching to promote the healthy development of university rhythmic gymnastics for health promotion actively ([5], p.11).

Cloud platform, also called cloud computing platform, is an emerging business computing model. Generic cloud platforms provide computing, storage, and networking resources and capabilities exposed via open APIs for application developers and other parties to develop applications easily. The “cloud” in cloud computing can be colloquially understood as a collection of various types of resources that exist on a cluster of servers in a cloud data center. Based on a cloud platform, the concept and importance of double-precision teaching in philosophical teaching were analyzed, and a basic framework of online and offline intelligent teaching based on blockchain technology was constructed ([6], p.11823). According to the security and dispersity of blockchain, an accurate learning resource teaching model based on learner knowledge representation and teaching resources was proposed. For example, Dunn et al. ([7], p.127) suggested that teachers approach mathematical modeling through mathematizing the context. However, in the processing of teaching resources ([8], p.535), at this stage there are problems such as poor resource classification, confusion of different types of teaching resources, and lack of individualization, therefore studying a teaching resource classification method with better application effects ([9], p.445). We suggest a framework to support teachers' modeling activities and demonstrate these using examples.

At present, universities generally have professional teaching resource databases under construction or completed ([10], p.33). However, many of these professional teaching resource databases are private systems that can only serve the users of the university, resulting in low resource utilization and repeated construction of various schools. Cloud computing ([11], p.25) has brought new opportunities for the construction of educational informatization. Suppose cloud computing technology can be introduced and establish a shared professional teaching resource library based on cloud computing. In that case, the co-construction and sharing of resource banks can be realized to a greater extent, the effect of resource classification can be improved, the reform of teaching methods and the improvement of teaching quality can be effectively promoted, and the balanced development can be effectively promoted. The teaching levels of the same type of school complement each other to better realize educational equity ([12], p.123).

The objective of our study was to solve the problems of low accuracy, low recall, and low F-measure value of classification results in traditional methods ([13], p.26). Thus, personalized rhythmic gymnastics for health promotion teaching resource classification algorithm based on cloud computing is proposed. Before the emergence of cloud computing technology, there were some difficult problems in constructing and using traditional professional teaching resource databases, such as low intelligence and lack of interactive and personalized services ([14], p.101). To provide personalized and high-level digital teaching resource library services, we suggest that additional hardware and software platforms must be built for users.

In sum, our study will contribute to solving the existing problem of rhythmic gymnastics resources. More specifically, the algorithm solves the problem of too high resource dimension and reduces the resource classification time and improves the classification accuracy ([15], p121). In addition, this study establishes a personalized rhythmic gymnastics for health promotion teaching resource database through cloud computing technology, records, arranges, and analyzes the teaching resources, provides personalized services for users, and provides technical support for the classification of teaching resources.

## 2. Literature Review

Interest in resource classification method based on cloud computing has increased attention from academics. Existing literature proposed a distributed resource space text classification model based on multielement neural network fusion and designed a multielement neural network path including word embedding layer, convolution layer, two-way gating cycle unit layer, attention mechanism layer, and softmax layer ([16], p.161). On this basis, the demand effect resource classification strategy is adopted to complete the mapping transformation from the demand of qualitative science and technology resources to the solution of quantitative resource service effect and then to the output of qualitative science and technology resources, focusing on the diversity of local and global semantic features of distributed science and technology resources and the significant long-distance dependence of text, and it is difficult to identify important resource information accurately ([17], p.12). Finally, the effect knowledge is quickly and accurately obtained from the distributed science and technology resource space to complete the text classification. Experiments verify the feasibility and effectiveness of this method, which provides a new idea and means for more comprehensive mining of resource text features, but this method has the problem of low accuracy of text classification. Aiming at the influence of new words in feature items on classification results, Ye et al. proposed a network new word text classification method based on the improved TF-IDF algorithm ([18], p.104). New comments are recognized in text preprocessing, and the calculation formula of feature weight is changed in vector space model representation to realize text classification. The experimental results show that this method can achieve the purpose of feature dimension reduction and optimize the text classification results, but this method has the problem of low F-measure value. Moreover, Xiao et al. ([19], p.1079) proposed a multi-label text classification method based on label semantic attention, which depends on the document's text and the corresponding label and shares words between the document and the label ([20], p.68). For document embedding, two-way long-term and short-term memory is used to obtain the implicit representation of each word, and the weight of each word in the document is obtained using the tag semantic attention mechanism to consider the importance of each word to the current tag. In addition, tags are often interrelated in semantic space. The semantic information of tags is used, and the relevance of tags is also considered ([21], p.51). Experimental results show that this method can effectively capture important words and realize the effective classification of multi-label text, but this method has the problem of low recall.

## 3. Methodology

### 3.1. Library Model Based on Cloud Computing

The personalized rhythmic gymnastics for health promotion teaching resource library based on cloud computing is a professional teaching data resource platform whose scale can be expanded as needed. It has a huge storage space and has the maintenance and safety guarantee of a professional technical team ([22], p.15). Users can use a variety of terminal devices to obtain the resources they need, or share them with other users ([23], p121). Because cloud computing is open and shared across devices and platforms, it makes it possible for large-scale data resources to be shared in the cloud. The cloud computing environment is a change in the technical environment for the personalized rhythmic gymnastics for health promotion teaching resource database. The corresponding changes must occur inside and outside the resource database to realize the transformation from traditional services to cloud services.  Figure 1 shows the overall architecture of personalized rhythmic gymnastics for health promotion teaching resource database based on cloud computing.

In the personalized rhythmic gymnastics for health promotion teaching resource library, the cloud layer of the resource library cloud service mode has an excellent infrastructure cluster, the first choice for large-scale storage of professional teaching resource library ([24], p.11). To build a professional teaching resource library based on cloud computing, it is necessary to set up basic equipment, cloud platforms, server-side applications, etc., in the cloud. These devices and systems in the cloud layer are centrally managed through the cloud management platform and provide services to the user side. In the user layer of resource library cloud service mode, users can realize the digital classroom of real-time resource sharing using wireless digital mobile devices. In the cloud computing environment, the personalized rhythmic gymnastics for health promotion teaching resource database has the ability to establish personal files for users. ([25], p.44). Collecting the characteristics and use preference information of users using the resource database establishes users' personalized use platform and work log and provides users with personalized services by recording, sorting, and analyzing these personalized behaviors.

### 3.2. Classification Algorithm Based on Distance-Weighted k-NN

Based on the personalized rhythmic gymnastics for health promotion teaching resource database established in Section 2, teaching resources are classified within the scope of the database. The main process of classification includes teaching resource preprocessing, teaching resource feature selection, teaching resource similarity calculation, and teaching resource classification four steps, through the above steps to output the classification results.

### 3.3. Preprocessing of Teaching Resources

First of all, the various types of artistic gymnastic teaching resources are preprocessed to determine the frequency of different resources. The calculation formula is as follows:

(1) $$\begin{array}{c} P_{n}=\sum_{i=\infty }^{\infty }{\left[x_{i}\left(m\right)-w_{i}\left(m\right)\right]}^{2}. \end{array}$$

The formula *x*_*i*_(*m*) represents the total number of occurrences in all resources; *w*_*i*_(*m*) represents the probability of resources appearing in a category; and *i* represents the total number of resources.

After obtaining the probability of all resources in various categories, all resource types are sorted according to categories, the top 500 resources are selected to join the statistical resource database, and then redundant resources are removed; that is, words that are meaningless to resource classification are removed. The specific removal method is to make an intersection of different types of resources, and the result of the intersection is regarded as the redundant part, which is removed from the statistical resources. Generally speaking, the number of resources in the statistical resource library should be controlled within 10000 resources.

500 teaching resources are taken as meta-samples. Generally speaking, meta-samples are defined as the linear combination of original samples, and meta-samples should contain the eigenstructure of resources. From another perspective, each teaching resource can be regarded as a linear combination of meta-samples. From a mathematical point of view, the teaching resource matrix *S* is decomposed into two matrices, namely *S*_*a*_ and *S*_*b*_. The relationship between the three is given as follows:

(2) $$\begin{array}{c} S=S_{a}+S_{b}. \end{array}$$

In the formula, both matrices *S*_*a*_ and *S*_*b*_ represent a teaching resource data set of *m* × *n*, each column represents a resource sample, and each row represents a characteristic of the resource. The size of matrix *S*_*a*_ is *m* × *l*, and each column in it is defined as a meta-sample; the size of matrix *S*_*b*_ is *l* × *n*. Each column represents the corresponding meta-sample expression mode, as shown in Figure 2.

Since the meta-sample contains the internal structure information of the training sample, this article uses the meta-sample instead of the sample in the training data set to preprocess the teaching resources. Meta-samples are extracted from each type of sample, and each type of teaching resource matrix is decomposed into two matrices:

(3) $$\begin{array}{c} S_{N}^{l}=S_{a}^{l}+S_{b}^{l}. \end{array}$$

In the formula, *S*_*a*_^*l*^ and *S*_*b*_^*l*^ represent the number of *l*th class element samples in the matrices *S*_*a*_ and *S*_*b*_, respectively. In practical applications, these two values are determined according to actual scenarios. This article uses the following formula to calculate the number of meta-samples:

(4) $$\begin{array}{c} L_{\text{total}}=\sum_{l=1}^{N}{\left|X\left(l\right)\right|}^{2}H_{i}\left(l\right). \end{array}$$

In the formula, *X*(*l*) represents the sparse coefficient of the meta-sample; *H*_*i*_(*l*) represents the query sample. After calculating the number of meta-samples, all the meta-samples are synthesized into the training data meta-sample set:

(5) $$\begin{array}{c} L=\left\{l_{1},l_{2},\ldots ,l_{N}\right\}. \end{array}$$

After preprocessing, the teaching resources of rhythmic gymnastics for health promotion still have problems such as high dimensionality and complex relevance. Therefore, the meta-sample set is further processed.

### 3.4. Feature Selection of Teaching Resources

Most of the massive original feature items have little effect on the classification results. The purpose of feature selection is to filter out the most powerful feature items from these massive original feature items for retention, to achieve the purpose of reducing the dimensionality of the high-dimensional feature vector space, reducing the amount of calculation in the subsequent classification process, and avoiding “the disaster of dimensionality.” This article takes the meta-sample set obtained in Section 3.1 as the object and mainly adopts the information gain method to select the characteristics of personalized rhythmic gymnastics for health promotion teaching resources.

Information gain is a feature selection method based on machine learning ([13], p.114820). The importance of the feature in the resource is determined by calculating the amount of information contained in a feature item. The more information a feature item contains, the more information the feature item contains. The more important it is, the less information it contains, and the less important the feature item is. Then, the amount of information contained in the personalized rhythmic gymnastics for health promotion teaching resource database based on cloud computing minus the information difference in the resource database without the feature item is the amount of information contained in the feature item. The amount of information here is expressed by entropy, and its calculation formula is as follows:

(6) $$\begin{array}{c} T\left(L\right)=\sqrt{\frac{\int_{0}^{\omega }\left(\omega -\omega_{i}\right){\left|L\left(\omega \right)\right|}^{2}}{\int_{0}^{\omega }{\left|L\left(\omega \right)\right|}^{2}\left(\mu_{t}-\mu_{h}\right)}}. \end{array}$$

*ω* represents the feature item; *ω*_*i*_ represents the probability of the feature item in the resource library; *L*(*ω*) represents the resource probability with feature item *ω*; *μ*_*t*_ represents the probability that the resource sample contains the feature item; and *μ*_*h*_ represents the probability that the resource sample does not contain the feature item.

Information gain is a very effective feature selection method at present, but this method considers the absence of feature words as a case. Although it sometimes brings benefits to classification, in most cases, the interference to resource category determination is greater than its benefits.

Therefore, it is necessary to obtain the feature vector of the category by constructing the feature vector of each resource that determines the classification. The feature vector must undergo normalization processing. The definition of the normalization processing is as follows:

Let the feature vector set be *Z*={*z*_1_, *z*_2_,…, *z*_*m*_} and do the following processing for each feature vector *z*_*i*_ in it:

(7) $$\begin{array}{c} z_{i}=\frac{z_{i}}{Gz_{i}}. \end{array}$$

of which

(8) $$\begin{array}{c} Gz_{i}=\sum_{i=1}^{n}z_{i}^{2}\times T\;\left(L\right). \end{array}$$

The vector processed by formula (7) becomes a canonical eigenvector.

*z*_*i*_^*t*^ is taken as the feature vector of resource *t*, where 1 ≤ *i* ≤ *N*, and *z*_*i*_^2^ represents the weight of each feature in the resource set. The weight is related to two factors: the number of resource samples in the resource pool and the other is the location of resource samples.

According to the feature selection results obtained above, the dimension of the feature vector is further reduced to improve the accuracy of the classification results of educational resources.

Let *∂*_1_ and *∂*_2_, respectively, represent the dispersion matrix within and between classes, and the calculation formulas are as follows:

(9) $$\begin{array}{c} \partial_{1}=\left(\frac{a_{i}}{b_{j}}+1\right)\;\left(\frac{u}{\bar{e}}-m\right), \end{array}$$

(10) $$\begin{array}{c} \partial_{2}=\frac{\left[\alpha \lambda^{\left(1\right)}\left(j\right)+\beta \lambda^{\left(2\right)}\left(j\right)\right]}{\sum_{j=1}^{M}\left[\alpha \lambda^{\left(1\right)}\left(j\right)+\beta \lambda^{\left(2\right)}\left(j\right)\right]}. \end{array}$$

In the formula, *b*_*j*_ represents the total number of feature vectors of the category; *a*_*i*_ represents the total number of feature vectors in the category; and $\bar{e}$ represents the mean value of the feature vectors in the category.

If the intra-class dispersion matrix *∂*_1_ is non-singular, when *a*_*i*_ is the largest, there is a characteristic dimension:

(11) $$\begin{array}{c} W_{o}=\left|\frac{W^{T}\partial_{1}W}{W^{T}\partial_{2}W}\right|. \end{array}$$

In the formula, *W* represents the generalized eigenvectors of the interclass dispersion matrix and the intraclass dispersion matrix.

The characteristic vector of personalized rhythmic gymnastics for health promotion resource is processed by the following formula for dimensionality reduction:

(12) $$\begin{array}{c} W_{p}=\arg\underset{W}{\max}\left|W^{T}\partial_{i}W\right|. \end{array}$$

Through the above calculation, the dimensionality reduction processing result of the characteristic vector of the personalized rhythmic gymnastics for health promotion resource is obtained, which is helpful to improve the accuracy of the classification result of the educational resource.

### 3.5. Calculation of Similarity of Teaching Resources

According to the results of the feature selection of teaching resources, a vector space model is established to calculate the similarity of teaching resources ([26], p.607), to make up for the shortcomings of a single algorithm, and to improve the recall rate of the classification of personalized rhythmic gymnastics for health promotion teaching resources. According to the distribution characteristics of teaching resources, the inter-topic correlation value reflecting in-depth information is introduced, and the related resource collection is given by combining user query and correlation control threshold, and the vector space model is used to calculate the similarity of teaching resources.

The basic idea is as follows: for a resource in a collection of related resources, the more occurrences of the resource, the more relevant the resource is to the subject of operation; for a collection of related resources, the greater the number of occurrences of related resources, the more frequent the occurrence of the related resource. The resource is also more related to the operation theme; the more related resources in the operation theme collection appear, the more relevant the resource and the operation theme are. In terms of usage factors, the greater the click-through rate of the resource relative to the operation theme, the more relevant the resource and the operation theme. The detailed algorithm design is as follows.

Assuming that *U*_*ij*_ represents the semantic weight of related resources in resource *j* under the operating theme, the calculation formula is as follows:

(13) $$\begin{array}{c} \left\{\begin{array}{c} \sum_{i,j=1}^{N}\alpha_{r}\beta_{r}\left.\exp{\left\|w_{rj}\right\|}^{2}\right],\\ {\left\|w_{rj}\right\|}^{2}=w_{r}^{T}w_{j}^{T}. \end{array}\right.. \end{array}$$

In the formula, *α*_*r*_ represents the vector space; *β*_*r*_ represents the Boolean vector; *w*_*rj*_ represents the total number of resources under the operation theme; *w*_*r*_^*T*^ and *w*_*j*_^*T*^ both represent the total amount of resources under the operation theme. The occurrence of the operation topic in the resource is recorded as 1, and the absence of the operation topic is recorded as 0. In the resource classification, the initial value of the parameter is 0.1, which is adjusted according to the number of resources.

The similarity coefficient of various resources in the resource pool is defined as *D*_sim_, and its calculation formula is as follows:

(14) $$\begin{array}{c} D_{\text{sim}}=\frac{D_{a}}{1+E_{a}}. \end{array}$$

In the formula, *D*_*a*_ represents the characteristics of the resources in the operation theme set; *E*_*a*_ represents the contribution degree of the feature weight to the similarity of the resources.

### 3.6. Classification Algorithm

The k-NN classification algorithm ([27], p.241) is a classification method based on statistics. This method is for the resource *X* to be classified. First, the *k* neighbors that are most similar to the resource in the training set are found, and the categories of these *k* neighbors are used as candidate categories. Then, the category whose occurrence times exceed a certain threshold in the *k* neighbors is assigned to the resource to be classified. An improvement of this method is to use the distance-weighted k-NN algorithm, which uses the distance (or similarity) between *k* neighbors and the resource to be classified as the weight of the category to which the neighbor belongs to calculate the probability of each candidate category. Then, the categories whose occurrence probability exceeds a certain threshold are assigned to the resources to be classified ([28], p.6717).

This study uses the distance-weighted k-NN algorithm to classify individual rhythmic gymnastics for health promotion teaching resources ([29], p.367). When calculating the similarity between resource *X* and training set resource *x*_*d*_, the similarity coefficient obtained in the above text is used as the basis for all resources. It is expressed as a vector in a vector space with a feature as a dimension, and the cosine value of the angle between the vectors is used to calculate the similarity between resources. The specific formula is as follows:

(15) $$\begin{array}{c} Y\left(x_{d}\right)=\frac{c\times x_{d}}{\left\|c\right\|\times \left\|x_{d}\right\|}\times D_{\text{sim}}, \end{array}$$

where *c* represents the vector of the resource to be classified in the training set. The calculation formula for the probability that the resource to be classified appears in its nearest neighbor is as follows:

(16) $$\begin{array}{c} B_{k}=\sum_{k=1}^{N}\frac{\ln\;\left(r_{k}-n_{k}\right)}{\log\sqrt{{\left(f_{k}\right)}^{n}+1}}. \end{array}$$

In the formula, *r*_*k*_ represents the probability that the candidate category appears in its *k* neighbors; *n*_*k*_ represents the category to which the resource belongs in *k* neighbors; and (*f*_*k*_)^*n*^ represents the resource dimension.

According to the above analysis, through the four steps of teaching resource preprocessing, teaching resource feature selection, teaching resource similarity calculation, and teaching resource classification, this study not only realizes the purpose of reducing the amount of calculation but also improves the recall rate of personalized rhythmic gymnastics for health promotion teaching resource classification. The classification result output through the above steps is better.

## 4. Results and Discussion

To systematically study the performance of personalized rhythmic gymnastics for health promotion teaching resource classification algorithm based on cloud computing, especially its classification performance in the classification of different data sets, this study designs the following scheme to test and analyze the results of the algorithm.

### 4.1. Data Set

To be able to compare objectively with other classification methods, this article uses the standard text classification data set Reuters 21575 to test the cloud computing-based personalized rhythmic gymnastics for health promotion teaching resource classification algorithm. At the same time, to accurately understand and reflect the classification effect of the algorithm on artistic gymnastic teaching resources, the distributed resource spatial text classification model based on multi-neural network fusion and the network new word text classification method based on the improved TF-IDF algorithm are used as comparison methods. The classification performance of different methods is tested ([13], p.114820).

The category distribution of the data set used in this test is shown in Table 1, which gives the number of categories in which resources appear at least once and 20 times in the data set and the probability of belonging to a category when a certain type of resources is randomly classified according to the total number of categories.

The data set in Table 1 is taken as the experimental data and is classified. During the experiment, MATLAB software is used to process the experimental data to ensure the validity and accuracy of the experimental results.

### 4.2. Test Results and Analysis

To evaluate the classification performance of the algorithm in this study, the classification accuracy rate and the classification recall rate are used as evaluation indicators to compare different methods. The calculation formula of the two is as follows:

(17) $$\begin{array}{c} \text{precision}\left(v_{1},v_{2}\right)=\frac{n\left(v_{1}\right)}{n\left(v_{2}\right)}, \end{array}$$

(18) $$\begin{array}{c} \text{recall}\left(v_{1},v_{2}\right)=\frac{n\left(v_{1}v_{2}\right)}{N}. \end{array}$$

In the formula, *v*_2_ represents the number of resources contained in category *v*; *v*_1_ represents the actual number of artistic gymnastics teaching resources in category *v*.

According to formula (17) and formula (18), the classification results of different methods of teaching resources are calculated. Among them, the classification accuracy results are shown in Figure 3.

According to the analysis of Figure 3, with the change in iteration times, the classification accuracy of different methods has no obvious change trend. When the number of iterations is 4, the classification accuracy of the algorithm in this study is 77%, the classification accuracy of the classification method based on multivariate neural network fusion is 64%, and the classification accuracy of the classification method based on the improved TF-IDF algorithm is 56%. When the number of iterations is 8, the classification accuracy of this algorithm is 65%, the classification accuracy of the classification method based on multivariate neural network fusion is 23%, and the classification accuracy of the classification method based on the improved TF-IDF algorithm is 48%. The comparison of the above data shows that the classification result of personalized rhythmic gymnastics for health promotion teaching resources is more reliable.

Figure 4 shows the result of resource classification recall rate.

According to the analysis of Figure 4, the highest recall of the algorithm in this study is 77%, the highest recall of the classification method based on multielement neural network fusion is 64%, and the highest recall of the classification method based on the improved TF-IDF algorithm is 45%. Through comparison, it can be seen that the recall of the algorithm in this study is higher, indicating that the algorithm can process more resources in the classification of teaching resources, and the comprehensiveness of the processing results is improved.

Formulas (17) and (18) reflect two different aspects of classification quality. To comprehensively consider the two, this study uses F-measure to evaluate the classification effect. The larger the value, the better the classification effect. The calculation method of F-measure is as follows:

(19) $$\begin{array}{c} F-\text{measure}=\frac{2\times \text{precision}\left(v_{1},v_{2}\right)\times \text{recall}\left(v_{1},v_{2}\right)}{\text{precision}\left(v_{1},v_{2}\right)+\text{recall}\left(v_{1},v_{2}\right)}. \end{array}$$

The classification results of teaching resources of different methods are calculated according to formula (19) and shown in Figure 5.

Figure 5 shows the classification results obtained by the three classification methods. When the number of iterations is lower than 2, the F-measure value keeps increasing; when the number of iterations reaches 1, the F-measure of the two traditional methods gradually slows down; and when the number of iterations reaches 2, the F-measure of the algorithm in this study gradually slows down. It is not difficult to see from Figure 5 that the F-measure value of the algorithm in this study is higher than that of the other two methods, which fully demonstrates the effectiveness of the method in this study.

To further verify the effectiveness of this algorithm, 100 teaching resource managers and teaching resource users are selected to evaluate the classification method, which is expressed in quantitative form. The scores are divided into as follows: 60–69 points are qualified, 70–79 points are medium, 80–89 points are good, and more than 90 points are excellent. The classified evaluation results of teaching resources are shown in Table 2.

From the trial evaluation results in Table 2, it can be seen that the algorithm in this study has the highest score, and the scoring results are basically in the good and excellent range, followed by the classification method based on the improved TF-IDF algorithm. The evaluation results of this method are mostly good. The classification method based on the improved TF-IDF algorithm is the worst, and the evaluation result of this method is even worse, which is basically medium and good. This is because this algorithm can eliminate useless resources and false information in the resource database and calculate the similarity of teaching resources. Although there are many kinds of resources in the resource database, this algorithm can still effectively classify resources to get a higher evaluation score.

## 5. Conclusion

In terms of the theoretical implications, this study contributes to the literature on cloud computing by presenting the sport resource classification algorithm for health promotion. Prior study has paid little attention to teaching resources optimization ([8], p.535). Moreover, there is a dearth of research on the rhythmic gymnastics for health promotion teaching method, which needs to switch from traditional way to information-based method ([3], p.13). To broaden the knowledge in this stream, we suggest a framework to support teachers' modeling activities and demonstrate with examples.

Aiming at the problems of low accuracy, low recall, and low F-measure value of traditional classification results, personalized rhythmic gymnastics for health promotion teaching resource classification algorithm based on cloud computing is proposed. The experimental results fully verify the classification effectiveness of this algorithm. This algorithm solves the problem of too high resource dimension, reduces the resource classification time, and improves the classification accuracy. The experimental results show that the highest recall of this algorithm is 77%, which is much higher than the traditional methods, and the classification accuracy and F-measure value are high, which shows that this algorithm can effectively improve the effect of text classification. Although the proposed method has advantages in computational complexity, its recall rate is not high enough. In future works, we will refine models and expand data samples to improve recall rate.

## Figures and Tables

**Figure 1:** Overall structure of a personalized rhythmic gymnastics for health promotion teaching resource library based on cloud computing.

**Figure 2:** Schematic diagram of the meta-sample model.

**Figure 3:** Comparison of classification accuracy of different methods.

**Figure 4:** Comparison of recall rates of different methods.

**Figure 5:** F-measure comparison of different methods.

**Table 1:** Experimental data set.

Data set	The probability that a certain type of resource appears at least once	The probability that a certain type of resource appears at least 20 times	Probability of belonging to a certain category
1	94.3	70.2	67.4
2	81.2	59.1	79.9
3	75.3	63.0	81.5
4	90.1	74.2	42.0
5	88.6	80.1	74.2
6	74.1	58.3	70.9
7	83.4	61.9	84.9

**Table 2:** Classification and evaluation results of teaching resources.

Number of evaluators/person	The algorithm proposed in this article	Classification method based on multivariate neural network fusion	Classification method based on the improved TF-IDF algorithm
10	97	90	87
20	96	90	85
30	96	90	84
40	95	87	83
50	94	87	80
60	92	86	79
70	90	85	79
80	89	83	78
90	88	81	78
100	87	80	76

## Data Availability

The data used to support the findings of this study are available from the corresponding author upon request.
